# Value of Serum miR-34a and Ang-1 in Severity Evaluation and Prognosis of Neonatal Respiratory Distress Syndrome

**DOI:** 10.1155/2022/5480026

**Published:** 2022-09-21

**Authors:** Qiaoyu Li, Yongcun Chen, Liangfeng Lin

**Affiliations:** Department of Pediatrics, The Second Affiliated Hospital of Fujian Medical University, Quanzhou 362000, Fujian, China

## Abstract

**Methods:**

A total of 96 neonates with RDS admitted to the hospital from February 2020 to April 2021 were selected as the research subjects. According to the neonatal critical illness score, the subjects were divided into non-critical group (*n* = 50), critical group (*n* = 27), and extremely critical group (*n* = 19). According to survival status, the subjects were divided into survival group (*n* = 76) and death group (*n* = 20). Serum miR-34a and Ang-1 levels and NCIS were compared between RDS neonates with different severity and prognosis. The predictive value of serum miR-34a, Ang-1, and NCIS for death was analyzed using the receiver operating characteristic (ROC) curve.

**Results:**

Serum miR-34a and Ang-1 levels and NCIS were significantly different in the 3 groups (*P* < 0.05). Serum miR-34a level decreased in order, while serum Ang-1 level and NCIS increased in order from the extremely critical group, the critical group to the non-critical group (*P* < 0.05). The survival group had lower serum miR-34a level and higher Ang-1 level and NCIS than the death group (*P* < 0.05). ROC curve analysis showed that the area under the curve (AUC) values of serum miR-34a, Ang-1, and NCIS to predict death of RDS neonates were 0.745, 0.7667, and 0.736. The cutoff values were 1.175, 6.815 ng/mL, and 85 points. The AUC of joint prediction with the three was 0.924, significantly larger than that of each index. The sensitivity and specificity were 94.70% and 90.00%.

**Conclusion:**

Serum miR-34a, Ang-1, and NCIS are closely related to the severity and prognosis of neonatal RDS. Combined detection of the three is helpful for prognosis of neonatal RDS.

## 1. Introduction

Respiratory distress syndrome (RDS) is a type of disease with a high clinical mortality rate in pediatrics. The clinical manifestations of children are moaning, shortness of breath, purple and blue, etc. In severe cases, apnea, superficial breathing, and limb relaxation may occur. It is common in infants, and the younger the gestational age, the higher the incidence [1, 2]. The main cause of the disease is the reduction of primary or secondary alveolar surface material, which poses a great threat to the life and health of children [3]. At present, the pathogenesis of RDS is not yet clear clinically. It has been suggested that the lack of lung surface material and the imbalance of inflammatory response are the important pathological mechanisms of RDS [4]. MicroRNA (miRNA) is a gene regulatory molecule that regulates the immune response and inflammatory pathway by affecting the expression of target genes. In recent years, studies have shown that miR-34a can regulate the inflammatory response [5]. According to literature reports, different pathogenesis can increase the alveolar epithelial barrier and pulmonary vascular endothelial permeability in patients with RDS, and then pulmonary edema occurs. Angiopoietin (Ang) plays an important role in vascular endothelial proliferation and apoptosis [6, 7]. In view of this, this study detected serum miR-34a and Ang-1 levels in children with RDS and analyzed the value of these indicators in assessing the severity and prognosis of neonatal RDS.

## 2. Materials and Methods

### 2.1. General Information

A total of 96 children with RDS admitted to our hospital from February 2020 to April 2021 were selected as the research objects. Among them, there were 53 males and 43 females; the gestational age was 34–40 weeks, and the average gestational age was (37.07 ± 1.33) weeks. The birth weight was 2525g∼3370 g, and the average weight was (2950.54 ± 210.45) g. This study was approved by the Medical Theory Committee of the hospital, in accordance with the principles of the Declaration of Helsinki, and the patients and their families were informed and signed the consent form for this study.

Taking the diagnosis of RDS in children as the starting point of the study and taking the recovery and discharge or death as the end point of the study, all the children were divided into a survival group and a death group, with 76 cases and 20 cases, respectively. The Neonatal critical score (NCIS), which including heart rate, systolic blood pressure, respiration, and serum potassium of all children was performed [8]. Children with NCIS score >90 were classified as non-critical group, 70–90 were classified as critical group, and <70 were classified as extremely critical group, with 50 cases, 27 cases, and 19 cases, respectively.

### 2.2. Inclusion Criteria

Inclusion criteria were as follows: ① all children meet the relevant diagnostic criteria in Practical Neonatology [9]; ② the chest X-ray showed diffuse fine-grained reticular shadows, and the pulmonary transparency was reduced; and ③ the gestational age was over 34 weeks.

### 2.3. Exclusion Criteria

Exclusion criteria were as follows: ① combined with congenital pulmonary malformation, respiratory malformation, and so on; ② combined with severe extrapulmonary infection; and ③ combined with congenital complex heart disease.

### 2.4. Methods

#### 2.4.1. Serum miR-34a Detection

After diagnosis, 5 ml of morning venous blood was collected from all children, centrifuged to separate serum, and stored at −80°C for testing. 500 *μ*l serum was collected and allowed to stand with 1 mL of TRIzol at room temperature, isopropanol and 75% ethanol were added in turn, and the above operations were repeated to extract total RNA and store it at −20°C. The total RNA was reverse transcribed using a reverse transcription kit to synthesize cDNA products. The reaction system was 0.15 *μ*l dNTP (100 mmol/L), 1 *μ*l multi-stranded reversetranscriptase (50 U/*μ*l), 0.19 *μ*l lRNase inhibitor (20 U/*μ*l), and 4.16 *μ*l nuclease-free water, adding 5 *μ*l RNA solution (1.6 ng/*μ*l) and 3 *μ*l reverse transcription primers, mixing well, and centrifuging for 1 min. Cyclic reaction: 16°C for 30 minutes, 42°C for 30 minutes, 85°C for 5 minutes, ice bath for 1 minute, and stored at −20°C. Real-time fluorescence quantitative polymerase chain reaction was performed using a real-time fluorescence quantitative PCR instrument. Real-time fluorescence quantitative polymerase chain reaction (2 *μ*l cDNA, 3 *μ*l of upper and lower primers, and 0.5 *μ*l of Taq polymerase) was performed using real-time fluorescence quantitative PCR instrument. Reaction conditions: denaturation at 95°C for 15 s. After annealing at 60°C for 1 min, the reaction was terminated after 30 cycles of amplification, and the relative expression level of serum miR-34a was calculated by the 2^−ΔΔCt^ method.

#### 2.4.2. Detection of Ang-1 Level

The early morning venous blood was collected from the children and centrifuged at 3000 r/min for 10 min in a centrifuge, and the Ang-1 level was detected by enzyme-linked immunosorbent assay.

### 2.5. Statistical Indicators

In this study, SPSS19.0 was used for analysis and processing, the count data were described by (n(%)), and the *χ*^2^ test was used for comparison between groups. The measurement data conforming to the normal distribution are presented in $\left(\bar{x}\pm s\right)$, the *t*-test is used for comparison between groups, and the one-way analysis of variance is used between multiple groups. Receiver operating characteristic curve (ROC) was used to analyze the predictive value of serum miR-34a, Ang-1, and NCIS scores for death in children with RDS. *P* < 0.05 was the detection level.

## 3. Results

### 3.1. Comparison of Serum miR-34a and Ang-1 Levels and NCIS Scores in Children with RDS of Different Severity

There were significant differences in serum miR-34a and Ang-1 levels and NCIS scores among the three groups (*P* < 0.05), and miR-34a and Ang-1 levels and NCIS score of extremely critical group were lower than the other two groups (*P* < 0.05). The serum miR-34a level in the critical group was higher than that in the non-critical group, and the serum Ang-1 level and NCIS score were lower than those in the non-critical group (*P* < 0.05), as shown in Figures 1–3.

### 3.2. Comparison of Serum miR-34a and Ang-1 Levels and NCIS Scores in Children with RDS with Different Prognosis

The serum miR-34a level in the survival group was lower than that in the death group, and the Ang-1 level and NCIS score were higher than those in the death group, and the difference was statistically significant (*P* < 0.05), as shown in Figures 4–6.

### 3.3. The Serum Levels of miR-34a, Ang-1, NCIS Score, and the Three Combined Detection on the Predictive Value of Death of RDS Children

The results of ROC curve analysis showed that the areas under the line of serum miR-34a, Ang-1, and NCIS scores for predicting death in children with RDS were 0.745, 0.7667, and 0.736, and the critical values were 1.175, 6.815 ng/mL, and 85 points, respectively. The offline area of combined detection for predicting death in children with RDS was 0.924, which was significantly higher than that of single detection, and its sensitivity and specificity were 94.70% and 90.00%, respectively, as shown in Table 1 and Figure 7.

## 4. Discussion

RDS is the main cause of neonatal death. At present, there is still a lack of specific therapeutic methods for RDS, mainly through pulmonary surfactant replacement, respiratory support, fluid management, and other methods, and the treatment is difficult [10]. This disease has a poor prognosis and many sequelae, which pose a great threat to the life and health of children. Timely and effective prediction of the severity of the disease has positive significance for improving the prognosis and reducing the mortality rate of children. Serum miR-34a has been confirmed by studies to play an important role in cell proliferation, differentiation, and metabolism and is significantly related to immune inflammatory response [11]. Ang is a secretory endothelial cell-specific growth factor, mainly including Ang-1, Ang-2, Ang-3, Ang-4, and so on. Among them, Ang-1 and Ang-2 are more studied in inflammation, and studies have pointed out that monitoring the level of Ang-1 is helpful to evaluate the survival status of ARDS patients [12, 13].

Studies have confirmed that serum miR-34a plays an important role in cell proliferation, differentiation, and metabolism, and some studies have pointed out that it can be used as an effective index to evaluate the prognosis of RDS [14]. The results of this study showed that the level of serum miR-34a gradually increased with the aggravation of children's condition, and the level of serum miR-34a in critically ill recombinant children was higher than that in other two groups. It shows that the level of serum miR-34a is significantly correlated with the severity of the disease. In addition, the level of serum miR-34a in the survival group is lower than that in the death group, which suggests that serum miR-34 may be involved in the progress of neonatal RDS and can be used as a marker for prognosis evaluation of children with RDS. The reason is that mRNA plays an important regulatory role in RDS cell apoptosis and inflammation. The occurrence of RDS can lead to different degrees of inflammation in the body, leading to the increase of the level of miR-34a. Data show that miRNA can regulate gene transcription and expression, participate in macrophage polarization, and play an important role in the pathophysiological process of epithelial cells, endothelial cells, and macrophages [15]. Macrophages can effectively resist harmful substances in the immune process and can eliminate invading pathogens. They play an important role in alveoli and can prevent lung injury caused by extrapulmonary causes [16]. Therefore, the level of miR-34a is closely related to the pathological process of RDS. In addition, under the influence of lung epithelial cell injury, it can also stimulate the alveolar wall and capillary wall to release the level of miR-34a into blood circulation. Also, with the aggravation of RDS, this inflammatory stimulation will be more obvious.

This study showed that the serum Ang-1 level and NCIS score gradually decreased, and the serum Ang-1 level and NCIS score were lower than those of the other two groups (*P* < 0.05). The serum Ang-1 level of critically ill patients and NCIS score were lower than those of non-critically ill patients, suggesting that serum Ang-1 level and NCIS score were closely related to the severity of RDS in children. On the other hand, studies have pointed out that monitoring Ang-1 levels can help to evaluate the survival status of patients with ARDS. In this study, the serum miR-34a level of children in the survival group was lower than that in the death group, and the Ang-1 level and NCIS score were higher than those in the death group (*P* < 0.05), further confirming the above view. Ang-1 is a vascular growth factor secreted by a variety of cells, which plays a regulatory role in maintaining vascular permeability. In previous studies, the downregulation of Ang-1 expression was responsible for the decreased stability and increased permeability of pulmonary capillary endothelial cells in patients with ARDS [17]. The main reason was that Ang-1 could not only reduce the synthesis of nitric oxide (NO) by degrading bradykinin but also promote the generation of oxygen free radicals induced by oxidative stress to increase the decomposition of NO and aggravate the damage of pulmonary vascular endothelial cells [18]. NCIS score is a domestic neonatal critical illness score method, which is mainly used to analyze and observe blood gas analysis, vital signs, biochemical tests, and other indicators of children [19]. The literature has shown that NCIS score has a good prediction effect on the death of children with RDS [20]. In this study, the ROC curve was used to analyze the predictive value of single test of serum miR-34a, Ang-1, NCIS scores, and the combination of the three tests on the death of children with RDS. It was found that the offline area for predicting the death of children with RDS by the combination of the three tests was 0.930, which was significantly higher than that by the single test. The sensitivity and specificity were 90.00% and 96.10%, respectively, indicating that the combination of the above three indicators had high predictive value for the prognosis of children with RDS and could be used as an auxiliary method for clinical diagnosis.

In conclusion, serum miR-34a, Ang-1, and NCIS scores are closely related to the disease severity and prognosis of children with RDS, and the combined detection of the three has a high predictive value for the prognosis of children with RDS. It provides new clues for clinical treatment. However, the shortcomings of this study are that the sample sources are concentrated, the sample size is small, and it is a single-center study. Future large-scale, multi-center research is needed to further demonstrate the research results.

## Figures and Tables

**Figure 1:** Comparison of serum miR-34a in children with different severity of RDS.

**Figure 2:** Comparison of serum Ang-1 levels in children with different severity of RDS.

**Figure 3:** Comparison of NCIS scores in children with RDS of different severity.

**Figure 4:** Comparison of serum miR-34a in children with RDS with different prognosis.

**Figure 5:** Comparison of serum Ang-1 levels in children with RDS with different prognosis.

**Figure 6:** Comparison of NCIS scores in children with RDS with different prognosis.

**Figure 7:** ROC curve analysis of serum miR-34a, Ang-1, and NCIS scores alone and their combined detection to predict death in children with RDS.

**Table 1:** Predictive value of serum miR-34a, Ang-1, and NCIS scores individually and their combined detection on death in children with RDS.

Indexes	Area under the curve	Standard deviation	95% CI	*P*	Critical value	Sensitivity (%)	Specificity (%)
miR-34a	0.745	0.064	0.620∼0.870	0.001	1.175	72.40	70.00
Ang-1	0.667	0.063	0.543∼0.791	0.022	6.815pg/mL	59.20	75.00
NCIS scale	0.736	0.060	0.618∼0.853	0.001	85 scale	80.30	60.00
Joint detection of the three	0.924	0.042	0.842∼1.000	0.001	—	94.70	90.00

## Data Availability

The data can be obtained from the corresponding author upon reasonable request.

## References

[1] Raimondi F., Migliaro F., Corsini I. (2021). Lung ultrasound score progress in neonatal respiratory distress syndrome. *Pediatrics*.

[2] Dargaville P. A., Kamlin C. O. F., Orsini F. (2021). Effect of minimally invasive surfactant therapy vs sham treatment on death or bronchopulmonary dysplasia in preterm infants with respiratory distress syndrome: the OPTIMIST-A randomized clinical trial. *JAMA*.

[3] Reynolds P., Bustani P., Darby C. (2021). Less-Invasive surfactant administration for neonatal respiratory distress syndrome: a consensus guideline. *Neonatology*.

[4] Wheeler C. R., Smallwood C. D. (2020). 2019 Year in review: neonatal respiratory support. *Respiratory Care*.

[5] Ramaswamy V. V., More K., Roehr C. C., Bandiya P., Nangia S. (2020). Efficacy of noninvasive respiratory support modes for primary respiratory support in preterm neonates with respiratory distress syndrome: systematic review and network meta-analysis. *Pediatric Pulmonology*.

[6] Alhassen Z., Vali P., Guglani L., Lakshminrusimha S., Ryan R. M. (2021). Recent advances in pathophysiology and management of transient tachypnea of newborn. *Journal of Perinatology*.

[7] Huo M. Y., Mei H., Zhang Y. H., Liu C. Z., Hu Y. N., Song D. (2020). [Efficacy and safety of less invasive surfactant administration in the treatment of neonatal respiratory distress syndrome: a Meta analysis]. *Zhong Guo Dang Dai Er Ke Za Zhi*.

[8] Gupta B. K., Saha A. K., Mukherjee S., Saha B. (2020). Minimally invasive surfactant therapy versus InSurE in preterm neonates of 28 to 34 weeks with respiratory distress syndrome on non-invasive positive pressure ventilation-a randomized controlled trial. *European Journal of Pediatrics*.

[9] Cimino C., Saporito M. A. N., Vitaliti G. (2020). N-BiPAP vs n-CPAP in term neonate with respiratory distress syndrome. *Early Human Development*.

[10] Ray S. (2021). Neonate with persisting respiratory distress after resolution of pneumothorax. *Arch Dis Child Educ Pract Ed*.

[11] Oishi P., Fineman J. R. (2020). Equipoise and acumen in pediatric acute respiratory distress syndrome research. *American Journal of Respiratory and Critical Care Medicine*.

[12] Karmoker R. K., Mirza T. T., Hossain A. K. (2020). Influence of the interval between antenatal corticosteroid therapy and delivery on the incidence of respiratory distress syndrome in neonate. *Mymensingh Medical Journal*.

[13] Elfarargy M. S., Al-Ashmawy G. M., Abu-Risha S., Khattab H. (2021). Novel adjuvant therapy with zinc supplementation in neonatal respiratory distress syndrome. *Endocrine, Metabolic & Immune Disorders - Drug Targets*.

[14] Xu Y., Xu Y., Zhu Y. (2020). Macrophage miR-34a is a key regulator of cholesterol efflux and atherosclerosis. *Molecular Therapy*.

[15] Li S., Wei X., He J. (2021). The comprehensive landscape of miR-34a in cancer research. *Cancer and Metastasis Reviews*.

[16] Shi X., Kaller M., Rokavec M., Kirchner T., Horst D., Hermeking H. (2020). Characterization of a p53/miR-34a/CSF1R/STAT3 feedback loop in colorectal cancer. *Cellular and Molecular Gastroenterology and Hepatology*.

[17] Zhou J., Li Z., Wu T., Zhao Q., Zhao Q., Cao Y. (2020). LncGBP9/miR-34a axis drives macrophages toward a phenotype conducive for spinal cord injury repair via STAT1/STAT6 and SOCS3. *Journal of Neuroinflammation*.

[18] Liu P., Ryczko M., Xie X. (2021). New soluble angiopoietin analog of Hepta-ANG1 prevents pathological vascular leakage. *Biotechnology and Bioengineering*.

[19] Cai G. L., Yang Z. X., Guo D. Y., Hu C. B., Yan M. L., Yan J. (2021). Macrophages enhance lipopolysaccharide induced apoptosis via Ang1 and NF-*κ*B pathways in human umbilical vein endothelial cells. *Scientific Reports*.

[20] Cao S., Deng Q., Wang Y., Zhou Y., Zhou Q. (2021). Ultrasound-targeted microbubble destruction-mediated Ang1 gene transfection improves left ventricular structural and sympathetic nerve remodeling in canines with myocardial infarction. *Annals of Translational Medicine*.

